# Comparison of Different First-Line Systemic Therapies in Advanced Biliary Tract Cancer Based on Updated Random Controlled Trials: A Systematic Review and Network Meta-Analysis

**DOI:** 10.1155/2022/1720696

**Published:** 2022-09-09

**Authors:** Long Feng, Ying Wang, Haoqian Xu, Fengming Yi

**Affiliations:** ^1^Department of Oncology, Second Affiliated Hospital of Nanchang University, Nanchang 330006, China; ^2^Jiangxi Key Laboratory of Clinical and Translational Cancer Research, Nanchang 330006, China

## Abstract

**Methods:**

We searched PubMed, Web of Science, and Cochrane Library for abstracts and full-text articles published from database inception through May 2022. All the random controlled trials (RCTs) were assessed and collected as eligible studies. The primary outcome was overall survival (OS). The second outcome was progression-free survival (PFS).

**Results:**

Seventeen studies, including 3632 patients, were selected from 1361 records. In the network meta-analysis for OS, gemcitabine + cisplatin (GemCis) + cediranib (HR, 0.11; 95% CI, 0.00-2.88), GemCis+durvalumab (HR, 0.27; 95% CI, 0.06-1.29), and GemCis + merestinib (HR, 0.37; 95% CI, 0.03-4.36) showed the trend of OS benefit over standard treatment (GemCis), although there was no significant difference. GemCis, GemOxa, and gemcitabine+S1 (GemS1) did not differ when comparing OS. In the network meta-analysis for PFS, GemCis+merestinib (HR, 0.67; 95% CI, 0.54-0.83) and GemCis+durvalumab (HR, 0.22; 95% CI, 0.08-0.62) showed PFS benefit over standard treatment (GemCis) with a significant difference. GemCis, GemOxa, and GemS1 did not differ when comparing PFS.

**Conclusion:**

GemCis+durvalumab might be the most promising regimen for advanced BTC when considering OS and PFS. GemOxa and GemS1 could be alternative options for advanced BTC patients with nontolerance to GemCis.

## 1. Introduction

Biliary tract cancer (BTC) is a heterogeneous and aggressive malignancy that occurs in the epithelial cell of the biliary tree with varied epidemiology worldwide. The classification according to the anatomic structure includes intrahepatic cholangiocarcinoma (iCC), perihilar CCA (pCC), distal CCA (dCC), and gallbladder cancer(GC) [1, 2], and there are other classifications in terms of etiology, histology, or molecular patterns [1, 2]. The prognosis of BTC is extremely poor, with the 5-year survival rate being limited to 2%, as most patients are diagnosed at a late stage [3].

Surgical resection and transplantation are currently identified as curative approaches for BTC patients in the early stage. Systemic therapy is considered the mainstay treatment for patients with advanced BTC. When considering chemotherapy, the median overall survival (mOS) for the established regimens ranges from 6 months to 19 months [3]. Gemcitabine plus cisplatin (GemCis) represents the first-line standard of care regimen according to the ABC-02 randomized phase III study, with prolonged median OS from 8.1 months to 11.7 months when compared with gemcitabine monotherapy [4]. However, GemCis plus nab-paclitaxel presents the highest mOS with 19.2 months in an open-label, single-arm phase II trial [5], and there needs to be a head-to-head clinical trial to verify it. Other chemotherapeutic regimens include gemcitabine plus oxaliplatin (GemOxa) [6], gemcitabine plus S-1(GemS1) [7], and capecitabine plus oxaliplatin (XELOX) [8], also proved to be effective in first-line treatment for advanced or unresectable BTC.

Emerging therapeutic strategies include molecular targeted therapy and immunotherapy based on current evidence. Molecular targets include fibroblast growth factor receptor (FGFR), isocitrate dehydrogenase (IDH), RAS–RAF–MEK (MAP2K1)–ERK (MAPK3), HER2 (also known as ERBB2), DNA mismatch repair, and NTRK, which are shown to be the most promising treatments till now, whereas the targeted therapy is limited to a small number of patients with gene mutation or gene aberrant. Some trials are trying to explore the combination of chemotherapy and nonspecific molecular drugs or antibodies [9–11]. Trials on the use of immunotherapy in BTCs are limited. Nevertheless, many ongoing trials explore immunotherapy such as PD-1, PD-L1, and CTLA-4 antibodies [2]. A recent abstract posted in ASCO demonstrated that additional durvalumab (PD-L1 inhibitor) improved the outcome of gemcitabine-based chemotherapy for patients with advanced BTC [12].

Herein, we aim to compare the efficacy of different first-line treatment regimens for patients with advanced BTC and find out whether gemcitabine-based chemotherapy combined with targeted therapy or immunotherapy is the best option. Moreover, gemcitabine plus oxaliplatin and gemcitabine plus S1 are comparable to gemcitabine plus platinum, which might be alternative options for patients with nontolerate GemCis.

## 2. Methods

This study was according to the Preferred Reporting Items for Systematic Review and Meta-Analyses (PRISMA) statement. Informed consent did not need to be signed, as the current meta-analysis was not based on individual patient level.

### 2.1. Search Strategies and Selection Criteria

We searched PubMed, Web of Science, and Cochrane Library from database inception up through May 2022 for abstracts and full-text articles published about the first-line treatment for patients with advanced biliary duct cancer. Keywords included “advanced biliary/bile duct cancer/carcinoma”, “unresectable/metastatic biliary/bile duct cancer/carcinoma”, “cholangiocarcinoma”, “first line”, “systemic therapy”, and “systemic treatment” were used to search for the clinical trials. The authors (LF and YW) made an agreement after consensus-based discussions. Random controlled trials that compared the efficacy of different systemic treatments in advanced biliary duct cancer were collected. We excluded single-arm studies and locoregional therapy. We also excluded the duplicate publications or studies published in the same center with patient overlap.

Two reviewers (YW and FMY) independently assessed and extracted data from each study. The basic information of studies included author/publication year, country, cohort, patient number, gender distribution, age, Eastern Cooperative Oncology Group (ECOG), and primary tumor. The primary outcome was overall survival. The secondary outcome was progression-free survival.

### 2.2. Risk of Bias Assessment

The quality of the trials was assessed by the Cochrane risk of bias tool, which included the following domains: random sequence generation, allocation concealment, blinding, incomplete outcome data, and selective outcome reporting [13]. Two authors (HQX and FMY) assessed the studies independently and made a consensus after discussion.

### 2.3. Statistical Analysis

The statistical analysis was conducted using Stata software (version 16, Stata Corp. LP, College Station, TX, USA). Review Manager 5.3 software (Cochrane Collaboration, Oxford, UK) was used to assess the risk bias. The heterogeneity of direct evidence and indirect evidence was according to the inconsistency factor and the value of heterogeneity. Network meta-analyses (NMA) of different treatments were using a random-effects model. League tables were generated for back-transformed network estimates. Hazard ratios (HRs) and 95% confidence intervals (CI) were used to compare different treatments.

## 3. Results

### 3.1. Study Selection and Characteristics

Seventeen studies, including 3632 patients, were selected from 1361 records (Figure 1) [4, 6–12, 14–22]. The comparison of the studies included the following: GemCis vs. S1 Cisplatin (S1Cis); Gem vs. S1 vs. GemS1; GemS1 vs. S1; vandetanib vs. Gem+vandetanib vs. Gem; best supportive care (BSC) vs. fluorouracil+folinic (FUFA) vs. GemOxa; GemOxa vs. GemOxa+erlotinib; GemOxa+cetuximab vs. GemOxa; GemCis+cediranib vs. GemCis; oxaliplatin + irinotecan + infusional fluorouracil (FOLFIRINOX) vs. GemCis; GemCis+ramucirumab vs. GemCis+merestinib vs. GemCis; GemCis vs. GemS1; GemOxa vs. XELOX; GemOxa vs. GemOxa+erlotinib; GemS1 vs. Gem; Gem vs. GemCis; GemCis+durvalumab vs. GemCis; GemOxa vs. GemCis; and GemOxa+panitumumab vs. GemOxa. All the studies included were randomized controlled trials, with matched number of patients, gender distribution, and ECOG in each trial. However, there was a selection bias between different trials, such as primary tumor distribution between trials. The details of the studies are presented in Table 1 at the end of the manuscript.

When we consider the risk of bias, most of the studies have perfect random sequence generation, complete outcome data, and low reporting bias, whereas the allocation concealment and different treatments correlated with other agents that were easy to distinguish cause the impossible for blinding of participants and personnel for nearly all trails. Moreover, a small number of studies reported blinding of outcome assessment. The risk of bias is presented in Figure 2.

### 3.2. Network Meta-Analysis

The global inconsistency between different comparisons did not show any difference (*p* = 0.8428). The local and loop inconsistency demonstrated no differences between the trials (*p* > 0.05). The network plot showed that GemCis was the standard treatment with the largest node size, and GemOxa was ranked the second node size; most other studies compared the treatment differences between them. Moreover, we could conclude that the evidence of GemCis+durvalumab should be more confident as the large node size represented the big sample size recruited. Most other treatments were restricted to one or two comparisons with limited patients (Figure 3).

In the network meta-analysis for OS (Table 2), GemCis+cediranib (HR, 0.11; 95% CI, 0.00-2.88), GemCis+durvalumab (HR, 0.27; 95% CI, 0.06-1.29), and GemCis+merestinib (HR, 0.37; 95% CI, 0.03-4.36) showed the trend of OS benefit over standard treatment (GemCis), although there was no significant difference. However, the trials on GemCis+cediranib, and GemCis+merestinib were based on phase II studies with a limited number of participants, and the primary endpoints were not OS, which might cause the bias of the results. We could conclude that GemCis+durvalumab was an effective combination with confident evidence from the abstract posted [12], and we were looking forward to the final publication of the trial. The combination of different chemotherapeutic drugs did not show any difference when comparing OS; then, we concluded that GemOxa and GemS1 could be alternative treatments for GemCis. The ranking of different treatments according to surface under the cumulative ranking curve (SUCRA) was as follows (Table 3 and Figure 4): GemCis + cediranib, 86.1%; GemCis + durvalumab, 80.4%; GemCis + merestinib, 74.7%; GemOxa, 71.5%; GemOxa + erlotinib, 69.9%; XELOX, 68.3%; GemOxa + panitumumab, 63.6%; GemS1, 60.3%; GemCis, 60.2%; S1Cis, 58%; GemOxa + cetuximab, 51.8%; Gem, 38.7%; Gem + vandetanib, 38.5%; FOLFIRINOX, 34.5%; GemCis + ramucirumab, 28.5%; Vandetanib, 21.9%; BSC, 17.3%; FUFA, 17.3%; S1, 8.4%.

In the network meta-analysis for PFS (Table 4), there was a trial with insufficient result that we eliminated [19]. GemCis+merestinib (HR, 0.67; 95% CI, 0.54-0.83) and GemCis+durvalumab (HR, 0.22; 95% CI, 0.08-0.62) still showed PFS benefit over standard treatment (GemCis) with significant difference. However, as GemOxa + merestinib was based on a phase II study with a limited number of participants and negative PFS benefit. We believed that GemCis+durvalumab was an effective combination with confident evidence when considering PFS from the abstract [12]. GemOxa+erlotinib (HR, 0.07; 95%CI, 0.00-1.38) ranked as the highest SUCRA, whereas there was no significant PFS benefit in the study when compared to GemOxa alone. GemOxa+panitumumab (HR, 0.15; 95% CI, 0.01-4.37) and GemOxa+cetuximab (HR, 0.20; 95% CI, 0.01-3.57) were also ranked as the appropriate choices for patients with wild-type KRAS, although there was no significant difference between them. The combination of different chemotherapeutic drugs did not show any difference when comparing PFS. The ranking of different treatments according to SUCRA was as follows (Table 5, Figure 5): GemOxa+erlotinib, 91.2%; GemCis + durvalumab, 82.7%; GemOxa + panitumumab, 81.2%; GemOxa + cetuximab, 79%; XELOX, 76%; GemOxa, 69.5%; GemCis + cediranib, 66%; GemCis+merestinib, 64.2%; GemS1, 63.7%; GemCis, 51.9%; S1Cis, 50.5%; GemCis + ramucirumab, 49%; FOLFIRINOX, 37.1%; S1, 22.5%; Gem, 21.6%; FUFA, 13.9%; Gem + vandetanib, 13.3%; Vandetanib, 10.5%; BSC, 6.2%.

## 4. Discussion

BTC is a heterogeneous cancer with a poor prognosis, as over 70% of BTCs are diagnosed at the locally advanced or metastatic stage without curative treatment [23]. Systemic therapy, including cytotoxic chemotherapy, targeted therapy, and immunotherapy, is trying to prolong the life span of these patients, and some of the trials show encouraging results.

Since the phase III randomized study ABC-02 established the combination of gemcitabine and cisplatin as the standard of care first-line treatment for locally advanced or metastatic biliary tract cancers, which improved PFS and OS for advanced biliary cases, there was still another exploration on different combinations of cytotoxic chemotherapy. The representation was the combination of gemcitabine and oxaliplatin [6, 8, 20], which showed comparable effectiveness with GemCis. The two regimens demonstrated similar efficacy in BTC cases when considering OS and PFS in our study. The second combination was gemcitabine and S1 [7, 15, 19], which also demonstrated noninferiority to the GemCis regimen. Our study confirmed it. GemS1 should be considered a convenient standard of care option for patients with advanced BTC that did not need hydration. Moreover, the combination of oxaliplatin and capecitabine also showed significant noninferiority to GemOxa, and it could be an alternative first-line treatment of BCTs [8], and our study also confirmed it. Taken together, our study demonstrated that GemCis was the basic cytotoxic chemotherapy; GemOxa and GemS1 could be alternative cytotoxic chemotherapeutics for patients with advanced BTCs.

However, there was still a long way to reach an expected overall survival for these patients. Although numerous targeted therapies focused on FGFR, IDH1, EGFR, HER2, VEGF, NTRK, BRAF, and MEK, some demonstrated encouraging effectiveness [3]. Nevertheless, these molecular or antibodies targeted specific genes or receptors, restricting their application in limited patients. There were some trials on targeted therapy with nonspecific genes, including vandetanib [9], erlotinib [16], cediranib [11], merestinib [18], ramucirumab [18], panitumumab [21], and cetuximab [10]. As the KRAS mutation was not common (<20%) [10], we recruited the trial one panitumumab [21] and cetuximab [10] in our study. Among them, the addition of erlotinib to gemcitabine and oxaliplatin showed the trend of extending the OS and PFS, confirmed by our research. Other tyrosine kinase inhibitors also demonstrated the trend of improving OS or PFS, but there should be more investigations to confirm them.

When it comes to immunotherapy, numerous ongoing trials were trying to explore the effectiveness of PD-1/PD-L1 in advanced BTCs [24–26], including immune monotherapy, immunotherapy plus targeted therapy, and immunotherapy plus cytotoxic chemotherapy. In a recent ASCO, Oh D-Y posted an encouraging result on PD-L1 antibody durvalumab plus GemCis for advanced BTC cases. It showed improvement in OS and PFS when compared to GemCis. Our study confirmed them; the durvalumab plus GemCis ranked as the most effective regimen compared to other combinations in both OS and PFS.

However, there were limitations in this NMA. Firstly, the primary sites of the BTC were not paired enough. For example, some trials included patients with more iCC or limited GBC. Secondly, the studies were designed differently with different allocation concealment and different blinding of participants and personnel, which impacted the results. Moreover, some treatment is a single-center trial with a limited number of patients recruited, which might restrict the application of the treatment.

In conclusion, first-line treatments' effectiveness in patients with advanced BTCs varies in trials. However, durvalumab plus GemCis shows promising improvement on OS and PFS, although it is reported by an abstract. GemCis remains the standard of care with moderate effectiveness on OS and PFS; GemOxa and GemS1 could be alternative options for patients with nontolerance to GemCis.

## Figures and Tables

**Figure 1:** PRISMA flow diagram of screening and selection strategy.

**Figure 2:** RCT bias was evaluated by the Cochrane risk of bias tool: (a) risk of bias summary; (b) risk of bias graph.

**Figure 3:** Network plot and funnel plot of studies included GemCis, gemcitabine plus cisplatin; GemOxa, gemcitabine plus oxaliplatin; GemS1, gemcitabine plus S-1; S1Cis, S1 plus cisplatin; XELOX, capecitabine plus oxaliplatin; BSC, best supportive care; FUFA, fluorouracil+folinic; and FOLFIRINOX, oxaliplatin plus irinotecan plus infusional fluorouracil.

**Figure 4:** Surface under the cumulative ranking curve for different regimens on overall survival. GemCis: gemcitabine plus cisplatin; GemOxa: gemcitabine plus oxaliplatin; GemS1: gemcitabine plus S-1; S1Cis: S1 plus cisplatin; XELOX: capecitabine plus oxaliplatin; BSC: best supportive care; FUFA: fluorouracil+folinic; FOLFIRINOX: oxaliplatin plus irinotecan plus infusional fluorouracil.

**Figure 5:** Surface under the cumulative ranking curve for different regimens on progression-free survival. GemCis: gemcitabine plus cisplatin; GemOxa: gemcitabine plus oxaliplatin; GemS1: gemcitabine plus S-1; S1Cis: S1 plus cisplatin; XELOX: capecitabine plus oxaliplatin; BSC: best supportive care; FUFA: fluorouracil+folinic; FOLFIRINOX: oxaliplatin plus irinotecan plus infusional fluorouracil.

**Table 1:** Baseline characteristics for patients included.

Author/Publication year	Country	Cohort	Number	Gender(M/F)	Age (years old)	ECOG	Primary tumor
Kang MJ, et al. [14]	Korea.	GemCis	49	31/18	59(32-77)	0-1:42(86%) 2:7(14%)	ICC:20(41%)ECC:29(59%)
		S1Cis	47	31/16	60(36-77)	0-1:43(91%) 2:4(9%)	ICC:18(38%)ECC:29(62%)

Li H, et al. [22]	China.	Gem	25	16/9	55.1±8.5	NR	NR
		S1	25	19/6	56.8±7.9	NR	NR
		GemS1	25	19/6	57.0±7.2	NR	NR

Morizane C, et al. [15]	Japan.	GemS1	51	27/24	66.0(39-78)	0:39(76.5%) 1:12(23.5%)	ICC:20(39.2%)CC:9(17.6%)GC:19(37.3%)AV:3(5.9%)
		S1	50	28/22	62.5(49-79)	0:37(74.0%) 1:13(26.0%)	ICC:20(39.2%)ECC:9(17.6%)GC:19(37.3%)AV:3(5.9%)

Santoro A, et al. [9]	Italy.	Vandetanib	59	25/34	62.4±10.1	0:38(64.4%) 1:20(33.9%) 2:1(1.7%)	ICC:27(45.8%)ECC:16(27.1%)GC:11(18.6%)AV:5(8.5%)
		Gem+Vandetanib	58	31/27	64.4±9.5	0:36(61.0%) 1:20(33.9%) 2:3(5.1%)	ICC:31(53.4%)ECC:10(17.3%)GB:13(22.4%)AV:4(6.9%)
		Gem	56	25/31	64.0±8.8	0:34(61.8%) 1:20(36.4%) 2:1(1.8%)	ICC:29(52.7%)ECC:13(22.4%)GC:7(12.7%)AV:6(10.9%)

Sharma A, et al. [6]	India.	BSC	27	6/21	Median:51	≤2:27(100%)	GC:27(100%)
		FUFA	28	5/23	Median:47	≤2:28(100%)	GC:28(100%)
		GemOxa	26	5/21	Median:49	≤2:26(100%)	GC:26(100%)

Lee J, et al. [16]	Korea.	GemOxa	133	79/54	61(55-68)	0:20(15%) 1:100(75%) 2:13(10%)	CC:84(63%)GC:47(35%)AV:2(2%)
		GemOxa+Erlotinib	135	91/44	59(54-66)	0:26(19%) 1:104(77%) 2:5(4%)	CC:96(71%)GC:35(26%)AV:4(3%)

Malka D, et al. [10]	France. Germany.	GemOxa+Cetuximab	76	43/33	61(35-75)	0:35(46%)1:36(47%)2:0(0%)Unspecified:5(7%)	CC:62(82%)GC:11(14%)AV:1(1%)Multifocal:1(1%)Unspecified:1(1%)
		GemOxa	74	42/32	62(39-75)	0:27(36%) 1:42(57%) 2:1(1%) Unspecified:4(5%)	CC:61(82%)GC:11(15%)AV:0(0%)Multifocal:1(1%)Unspecified:1(1%)

Valle JW, et al. [11]	UK.	GemCis+Cediranib	62	34/28	68.0(60.4-73.0)	0:27(44%) 1:35(56%)	ICC:14(23%)ECC:24(39%)GC:20(32%)AV:4(6%)
		GemCis	62	28/34	64.5(59.7-73.1)	0:28(45%) 1:34(55%)	ICC:15(24%)ECC:24(39%)GC:19(31%)AV:4(6%)

Phelip JM, et al. [17]	France.	FOLFIRINOX	94	57/37	65(58-70)	0:45(47.9%) 1:48(52.1%)	ICC:60(63.8%)ECC:18(19.1%)GC:16(17.1%)
		GemCis	96	47/49	63(55-67)	0:46(47.9%) 1:50(52.1%)	ICC:59(61.5%)ECC:20(20.8%)GC:17(17.7%)

Valle JW, et al. [18]	UK.	GemCis+Ramucirumab	106	46/60	64(58-71)	0:45(43%) 1:58(55%) Missing:3(2%)	ICC:56(53%)GC:24(23%)ECC:18(17%)AV:8(8%)
		GemCis+Merestinib	102	48/54	62(56-67)	0:52(51%) 1:50(49%) Missing:0(0%)	ICC:60(59%)GC:22(22%)ECC:14(14%)AV:6(6%)
		GemCis	101	53/48	59(52-68)	0:61(60%) 1:39(39%) Missing:1(1%)	ICC:55(55%)GC:26(26%)ECC:14(14%)AV:5(5%)

Morizane C, et al. [7, 26]	Japan.	GemCis	175	99/76	67(41-78)	0:130(74%) 1:45(26%)	GC:68(39%)ICC:50(29%)ECC:49(28%)AV:7(4%)
		GemS1	179	97/82	67(27-79)	0:124(69%) 1:55(31%)	GC:69(39%) ICC:44(25%) ECC:59(33%) AV:6(3%)

Kim ST, et al. [8]	Korea.	GemOxa	114	70/44	64.0(35.0-83.0)	0:25(22%) 1:86(75%) 2:3(2%)	CC:84(74%) GC:30(26%)
		XELOX	108	74/34	62.0(28.0-84.0)	0:35(32%) 1:71(66%) 2:1(1%)	CC:77(71%)GC:31(29%)

Sasaki T, et al. [19]	Japan.	GemS1	30	16/14	68(47-83)	0:18(60%) 1:11(37%) 2:1(3%)	GC:16(53%)ICC:8(27%)ECC:6(20%)
		Gem	32	20/12	75(55-86)	0:18(56%) 1:12(38%) 2:2(6%)	GC:14(44%)ICC:8(25%)ECC:10(31%)

Valle J, et al. [4]	UK.	Gem	206	98/108	63.2(23.4-84.8)	0:64(31.1%) 1:117(56.8%)2:24(11.7%)	GC:76(36.9%)CC:119(57.8%)AV:11(5.3%)
		GemCis	204	96/108	63.9(32.8-81.9)	0:66(32.4%) 1:111(54.4%) 2:27(13.2%)	GC:73(35.8%)CC:122(59.8%)AV:9(4.4%)

Oh DY, et al.2022 [12]	Multiple counties	GemCis+Durvalumab	341	169/172	64(20-84)	0:50.7%	NR
		GemCis	344	176/168	64(31-85)	0:47.4%	NR

Sharma A, et al. [20]	India.	GemOxa	119	43/76	48.1±9.92	0:7(5.9%)1:72(60.5%)2:40(33.6%)	GC:119(100%)
		GemCis	124	39/85	47.8±12.05	0:7(5.6%)1:64(51.6%)2:53(42.7%)	GC:124(100%)

Leone F, et al. [21]	Italy.	GemOxa+Panitumumab	45	17/28	63.9(46.7-78.5)	0-1:45(100%)	ICC: 21 (46.7%)ECC: 21 (26.7%)GC: 12 (26.6%)
		GemOxa	44	15/29	64.2(36.8-78.5)	0-1:43(97.7%)2:1(2.3%)	ICC: 21 (47.7%)ECC: 7 (15.9%)GC: 16 (36.4%)

GemCis, gemcitabine plus cisplatin; GemOxa, gemcitabine plus oxaliplatin; GemS1, gemcitabine plus S-1; S1Cis, S1 plus Cisplatin; XELOX, capecitabine plus oxaliplatin; BSC, best supportive care; FUFA, Fluorouracil+folinic; FOLFIRINOX, Oxaliplatin plus irinotecan plus infusional fluorouracil; iCC, intrahepatic cholangiocarcinoma; eCC, extrahepatic cholangiocarcinoma; pCC, perihilar cholangiocarcinoma; dCC, distal cholangiocarcinoma; GC, gallbladder cancer; AV, ampulla of Vater; NR, not report.

**Table 2:** League table of network meta-analysis for overall survival.

XELOX	0.01 (0.00,41.97)	0.33 (0.00,241.23)	0.00 (0.00,0.95)	0.04 (0.00,241.27)	0.37 (0.00,146.43)	0.61 (0.00,1354.88)	0.82 (0.00,321.73)	0.20 (0.00,203.30)	0.82 (0.00,165.96)	0.03 (0.00,14.67)	1.11 (0.00,533.95)	1.49 (0.00,530.77)	3.67 (0.01,2527.53)	0.41 (0.00,117.26)	0.09 (0.00,35.58)	0.01 (0.00,4.36)	0.05 (0.00,35.98)	0.01 (0.00,5.20)
153.84 (0.02,993240.63)	Vandetanib	51.26 (0.03,92246.31)	0.36 (0.00,246.30)	6.48 (0.06,682.50)	57.51 (0.08,39854.70)	93.31 (0.01,715102.88)	125.95 (0.07,227252.61)	31.06 (0.01,120941.94)	125.95 (0.12,135655.52)	5.14 (0.00,5983.74)	170.21 (0.13,215049.52)	229.74 (0.24,223152.33)	565.07 (0.33,972537.06)	62.61 (0.08,50881.98)	13.83 (0.02,8480.31)	0.94 (0.00,2748.49)	7.67 (0.00,13762.77)	0.85 (0.00,3124.77)
3.00 (0.00,2172.54)	0.02 (0.00,35.10)	S1Cis	0.01 (0.00,0.35)	0.13 (0.00,197.64)	1.12 (0.02,52.99)	1.82 (0.00,1653.10)	2.46 (0.02,285.55)	0.61 (0.00,219.90)	2.46 (0.05,120.36)	0.10 (0.00,5.63)	3.32 (0.05,215.00)	4.48 (0.11,181.68)	11.02 (0.10,1188.14)	1.22 (0.04,35.14)	0.27 (0.01,12.95)	0.02 (0.00,4.42)	0.15 (0.00,17.23)	0.02 (0.00,5.55)
432.41 (1.05,177966.17)	2.81 (0.00,1945.93)	144.09 (2.83,7345.30)	S1	18.22 (0.03,10727.31)	161.64 (56.25,464.50)	262.27 (0.50,138215.56)	354.03 (6.91,18140.78)	87.30 (0.46,16733.89)	354.03 (20.83,6016.86)	14.45 (0.71,295.87)	478.42 (19.38,11809.25)	645.76 (49.54,8417.50)	1588.30 (33.94,74324.37)	175.99 (22.83,1356.60)	38.89 (11.08,136.52)	2.64 (0.02,319.01)	21.55 (0.42,1093.41)	2.39 (0.01,418.21)
23.73 (0.00,135855.92)	0.15 (0.00,16.24)	7.91 (0.01,12357.14)	0.05 (0.00,32.31)	Gem+Vandetanib	8.87 (0.02,5227.58)	14.39 (0.00,98040.73)	19.43 (0.01,30443.90)	4.79 (0.00,16419.48)	19.43 (0.02,17980.72)	0.79 (0.00,794.48)	26.25 (0.02,28602.97)	35.44 (0.04,29509.32)	87.16 (0.06,130167.20)	9.66 (0.01,6700.38)	2.13 (0.00,1108.80)	0.14 (0.00,371.42)	1.18 (0.00,1843.55)	0.13 (0.00,423.85)
2.68 (0.01,1047.89)	0.02 (0.00,12.05)	0.89 (0.02,42.11)	0.01 (0.00,0.02)	0.11 (0.00,66.44)	GemS1	1.62 (0.00,815.43)	2.19 (0.05,104.01)	0.54 (0.00,97.82)	2.19 (0.14,33.46)	0.09 (0.00,1.66)	2.96 (0.13,66.51)	4.00 (0.34,46.27)	9.83 (0.23,425.34)	1.09 (0.16,7.22)	0.24 (0.07,0.85)	0.02 (0.00,1.85)	0.13 (0.00,6.27)	0.01 (0.00,2.44)
1.65 (0.00,3682.94)	0.01 (0.00,82.14)	0.55 (0.00,498.95)	0.00 (0.00,2.01)	0.07 (0.00,473.29)	0.62 (0.00,309.74)	GemOxa+Panitumumab	1.35 (0.00,680.47)	0.33 (0.00,416.10)	1.35 (0.01,361.54)	0.06 (0.00,30.89)	1.82 (0.00,1120.36)	2.46 (0.01,1127.17)	6.06 (0.01,5236.74)	0.67 (0.00,251.27)	0.15 (0.00,75.24)	0.01 (0.00,9.02)	0.08 (0.00,74.42)	0.01 (0.00,10.66)
1.22 (0.00,479.97)	0.01 (0.00,14.33)	0.41 (0.00,47.30)	0.00 (0.00,0.14)	0.05 (0.00,80.66)	0.46 (0.01,21.68)	0.74 (0.00,373.45)	GemOxa+Erlotinib	0.25 (0.00,44.83)	1.00 (0.07,15.38)	0.04 (0.00,2.31)	1.35 (0.02,87.98)	1.82 (0.04,74.39)	4.49 (0.04,485.90)	0.50 (0.02,14.40)	0.11 (0.00,5.30)	0.01 (0.00,0.85)	0.06 (0.00,7.05)	0.01 (0.00,1.12)
4.95 (0.00,4987.37)	0.03 (0.00,125.37)	1.65 (0.00,599.01)	0.01 (0.00,2.20)	0.21 (0.00,715.36)	1.85 (0.01,335.33)	3.00 (0.00,3755.34)	4.06 (0.02,737.14)	GemOxa+Cetuximab	4.06 (0.05,339.33)	0.17 (0.00,34.15)	5.48 (0.02,1259.63)	7.40 (0.05,1197.72)	18.19 (0.05,6238.61)	2.02 (0.02,255.77)	0.45 (0.00,81.61)	0.03 (0.00,10.81)	0.25 (0.00,89.31)	0.03 (0.00,13.29)
1.22 (0.01,247.58)	0.01 (0.00,8.55)	0.41 (0.01,19.94)	0.00 (0.00,0.05)	0.05 (0.00,47.64)	0.46 (0.03,6.97)	0.74 (0.00,198.42)	1.00 (0.07,15.38)	0.25 (0.00,20.63)	GemOxa	0.04 (0.00,0.79)	1.35 (0.06,31.76)	1.82 (0.15,22.36)	4.49 (0.10,201.55)	0.50 (0.07,3.54)	0.11 (0.01,1.72)	0.01 (0.00,0.36)	0.06 (0.00,2.97)	0.01 (0.00,0.51)
29.93 (0.07,13137.47)	0.19 (0.00,226.47)	9.97 (0.18,560.41)	0.07 (0.00,1.42)	1.26 (0.00,1263.82)	11.19 (0.60,207.33)	18.15 (0.03,10177.44)	24.50 (0.43,1384.65)	6.04 (0.03,1246.77)	24.50 (1.26,476.38)	GemCis+Ramucirumab	33.11 (3.43,320.12)	44.70 (2.96,674.73)	109.93 (2.13,5682.62)	12.18 (1.32,112.61)	2.69 (0.14,50.92)	0.18 (0.00,23.94)	1.49 (0.03,83.43)	0.17 (0.00,31.21)
0.90 (0.00,436.18)	0.01 (0.00,7.42)	0.30 (0.00,19.50)	0.00 (0.00,0.05)	0.04 (0.00,41.49)	0.34 (0.02,7.59)	0.55 (0.00,336.68)	0.74 (0.01,48.17)	0.18 (0.00,41.94)	0.74 (0.03,17.39)	0.03 (0.00,0.29)	GemCis+Merestinib	1.35 (0.07,25.04)	3.32 (0.06,198.32)	0.37 (0.03,4.36)	0.08 (0.00,1.86)	0.01 (0.00,0.81)	0.05 (0.00,2.90)	0.00 (0.00,1.05)
0.67 (0.00,237.99)	0.00 (0.00,4.23)	0.22 (0.01,9.05)	0.00 (0.00,0.02)	0.03 (0.00,23.50)	0.25 (0.02,2.90)	0.41 (0.00,185.93)	0.55 (0.01,22.36)	0.14 (0.00,21.89)	0.55 (0.04,6.72)	0.02 (0.00,0.34)	0.74 (0.04,13.75)	GemCis+Durvalumab	2.46 (0.07,91.03)	0.27 (0.06,1.29)	0.06 (0.01,0.71)	0.00 (0.00,0.41)	0.03 (0.00,1.35)	0.00 (0.00,0.55)
0.27 (0.00,187.33)	0.00 (0.00,3.05)	0.09 (0.00,9.78)	0.00 (0.00,0.03)	0.01 (0.00,17.13)	0.10 (0.00,4.41)	0.17 (0.00,142.79)	0.22 (0.00,24.14)	0.05 (0.00,18.85)	0.22 (0.00,10.01)	0.01 (0.00,0.47)	0.30 (0.01,17.99)	0.41 (0.01,15.05)	GemCis+Cediranib	0.11 (0.00,2.88)	0.02 (0.00,1.08)	0.00 (0.00,0.38)	0.01 (0.00,1.46)	0.00 (0.00,0.48)
2.46 (0.01,707.90)	0.02 (0.00,12.98)	0.82 (0.03,23.55)	0.01 (0.00,0.04)	0.10 (0.00,71.84)	0.92 (0.14,6.09)	1.49 (0.00,558.03)	2.01 (0.07,58.26)	0.50 (0.00,62.94)	2.01 (0.28,14.34)	0.08 (0.01,0.76)	2.72 (0.23,32.19)	3.67 (0.77,17.40)	9.03 (0.35,234.78)	GemCis	0.22 (0.03,1.51)	0.01 (0.00,1.15)	0.12 (0.00,3.50)	0.01 (0.00,1.56)
11.12 (0.03,4399.84)	0.07 (0.00,44.31)	3.71 (0.08,177.81)	0.03 (0.01,0.09)	0.47 (0.00,243.48)	4.16 (1.18,14.67)	6.74 (0.01,3422.44)	9.10 (0.19,439.12)	2.25 (0.01,411.33)	9.10 (0.58,142.17)	0.37 (0.02,7.03)	12.30 (0.54,281.90)	16.61 (1.40,197.13)	40.84 (0.93,1796.71)	4.53 (0.66,30.97)	Gem	0.07 (0.00,7.81)	0.55 (0.01,26.47)	0.06 (0.00,10.27)
163.91 (0.23,117113.23)	1.07 (0.00,3120.00)	54.62 (0.23,13199.07)	0.38 (0.00,45.84)	6.91 (0.00,17720.67)	61.27 (0.54,6962.16)	99.41 (0.11,89151.14)	134.20 (1.18,15315.42)	33.09 (0.09,11835.69)	134.20 (2.80,6429.06)	5.48 (0.04,717.97)	181.35 (1.23,26745.98)	244.78 (2.44,24591.10)	602.05 (2.65,136883.86)	66.71 (0.87,5112.90)	14.74 (0.13,1696.22)	FUFA	8.17 (0.03,1967.45)	0.91 (0.02,39.51)
20.06 (0.03,14484.18)	0.13 (0.00,234.11)	6.69 (0.06,770.32)	0.05 (0.00,2.35)	0.85 (0.00,1318.04)	7.50 (0.16,352.59)	12.17 (0.01,11022.15)	16.43 (0.14,1901.68)	4.05 (0.01,1465.57)	16.43 (0.34,800.83)	0.67 (0.01,37.50)	22.20 (0.34,1431.03)	29.96 (0.74,1208.56)	73.70 (0.69,7912.07)	8.17 (0.29,233.62)	1.80 (0.04,86.17)	0.12 (0.00,29.48)	FOLFIRINOX	0.11 (0.00,37.00)
181.03 (0.19,170284.88)	1.18 (0.00,4326.85)	60.32 (0.18,20202.81)	0.42 (0.00,73.30)	7.63 (0.00,24666.99)	67.67 (0.41,11183.92)	109.80 (0.09,128487.02)	148.21 (0.89,24602.12)	36.55 (0.08,17748.36)	148.21 (1.97,11142.27)	6.05 (0.03,1141.76)	200.29 (0.95,42193.50)	270.34 (1.83,39875.12)	664.94 (2.10,210244.08)	73.68 (0.64,8474.71)	16.28 (0.10,2722.17)	1.10 (0.03,48.19)	9.02 (0.03,3012.00)	BSC

GemCis: gemcitabine plus cisplatin; GemOxa: gemcitabine plus oxaliplatin; GemS1: gemcitabine plus S-1; S1Cis: S1 plus cisplatin; XELOX: capecitabine plus oxaliplatin; BSC: best supportive care; FUFA: fluorouracil+folinic; FOLFIRINOX: oxaliplatin plus irinotecan plus infusional fluorouracil.

**Table 3:** Surface under the cumulative ranking curve values for overall survival.

Treatment	SUCRA
GemCis+Cediranib	86.1
GemCis+Durvalumab	80.4
GemCis+Merestinib	74.7
GemOxa	71.5
GemOxa+Erlotinib	69.9
XELOX	68.3
GemOxa+Panitumumab	63.6
GemS1	60.3
GemCis	60.2
S1Cis	58
GemOxa+Cetuximab	51.8
Gem	38.7
Gem+Vandetanib	38.5
FOLFIRINOX	34.5
GemCis+Ramucirumab	28.5
Vandetanib	21.9
BSC	17.3
FUFA	17.3
S1	8.4

GemCis: gemcitabine plus cisplatin; GemOxa: gemcitabine plus oxaliplatin; GemS1: gemcitabine plus S-1; S1Cis: S1 plus cisplatin; XELOX: capecitabine plus oxaliplatin; BSC: best supportive care; FUFA: fluorouracil+folinic; FOLFIRINOX: oxaliplatin plus irinotecan plus infusional fluorouracil.

**Table 4:** League table of network meta-analysis for progression-free survival.

XELOX	0.00 (0.00,0.27)	0.17 (0.00,10.22)	0.02 (0.00,0.85)	0.00 (0.00,0.41)	0.37 (0.01,15.83)	1.49 (0.04,57.99)	3.00 (0.12,77.38)	1.11 (0.04,27.26)	0.61 (0.04,8.43)	0.20 (0.01,6.49)	0.33 (0.01,10.47)	1.00 (0.03,36.18)	0.41 (0.01,18.64)	0.22 (0.01,6.97)	0.01 (0.00,0.50)	0.00 (0.00,0.11)	0.07 (0.00,3.66)	0.00 (0.00,0.06)
304.78 (3.77,24666.12)	Vandetanib	50.51 (1.44,1769.22)	4.70 (0.17,132.63)	1.35 (0.10,17.38)	111.69 (5.17,2413.56)	454.67 (5.92,34913.49)	915.60 (16.77,49995.71)	336.83 (6.39,17758.75)	184.86 (5.48,6231.83)	61.70 (3.86,986.06)	101.72 (6.55,1580.73)	305.59 (16.52,5653.47)	124.24 (5.04,3060.64)	68.19 (4.42,1050.81)	4.18 (0.33,52.49)	1.25 (0.02,71.19)	20.54 (0.68,621.06)	0.62 (0.01,35.57)
6.03 (0.10,372.13)	0.02 (0.00,0.69)	S1Cis	0.09 (0.00,2.00)	0.03 (0.00,1.10)	2.21 (0.14,34.33)	9.00 (0.15,524.88)	18.13 (0.45,732.86)	6.67 (0.17,259.57)	3.66 (0.15,87.30)	1.22 (0.12,12.38)	2.01 (0.21,19.74)	6.05 (0.50,72.93)	2.46 (0.15,41.25)	1.35 (0.14,13.10)	0.08 (0.01,1.01)	0.02 (0.00,1.05)	0.41 (0.02,8.59)	0.01 (0.00,0.52)
64.85 (1.18,3567.02)	0.21 (0.01,6.00)	10.75 (0.50,230.59)	S1	0.29 (0.01,9.62)	23.77 (5.24,107.76)	96.74 (1.86,5023.05)	194.82 (5.48,6930.57)	71.67 (2.10,2451.33)	39.33 (1.92,807.39)	13.13 (1.60,107.85)	21.64 (2.73,171.34)	65.02 (6.55,645.40)	26.44 (1.87,374.05)	14.51 (1.85,113.59)	0.89 (0.10,7.86)	0.27 (0.01,9.92)	4.37 (0.24,78.96)	0.13 (0.00,4.96)
225.81 (2.45,20850.08)	0.74 (0.06,9.54)	37.42 (0.91,1540.78)	3.48 (0.10,116.66)	Gem+Vandetanib	82.75 (3.18,2153.07)	336.86 (3.84,29557.82)	678.36 (10.75,42794.08)	249.55 (4.09,15219.42)	136.96 (3.45,5436.28)	45.71 (2.33,896.40)	75.36 (3.94,1439.80)	226.41 (10.07,5090.31)	92.05 (3.13,2710.76)	50.52 (2.66,957.68)	3.10 (0.20,48.58)	0.92 (0.01,60.84)	15.22 (0.43,544.47)	0.46 (0.01,30.39)
2.73 (0.06,117.88)	0.01 (0.00,0.19)	0.45 (0.03,7.02)	0.04 (0.01,0.19)	0.01 (0.00,0.31)	GemS1	4.07 (0.10,165.37)	8.20 (0.30,221.87)	3.02 (0.12,78.22)	1.66 (0.11,24.46)	0.55 (0.11,2.73)	0.91 (0.19,4.29)	2.74 (0.43,17.25)	1.11 (0.12,10.74)	0.61 (0.13,2.83)	0.04 (0.01,0.21)	0.01 (0.00,0.32)	0.18 (0.01,2.35)	0.01 (0.00,0.16)
0.67 (0.02,26.06)	0.00 (0.00,0.17)	0.11 (0.00,6.48)	0.01 (0.00,0.54)	0.00 (0.00,0.26)	0.25 (0.01,9.98)	GemOxa+Panitumumab	2.01 (0.08,48.29)	0.74 (0.03,17.00)	0.41 (0.03,5.17)	0.14 (0.00,4.07)	0.22 (0.01,6.56)	0.67 (0.02,22.73)	0.27 (0.01,11.76)	0.15 (0.01,4.37)	0.01 (0.00,0.31)	0.00 (0.00,0.07)	0.05 (0.00,2.32)	0.00 (0.00,0.03)
0.33 (0.01,8.57)	0.00 (0.00,0.06)	0.06 (0.00,2.23)	0.01 (0.00,0.18)	0.00 (0.00,0.09)	0.12 (0.00,3.30)	0.50 (0.02,11.91)	GemOxa+Erlotinib	0.37 (0.03,5.16)	0.20 (0.03,1.36)	0.07 (0.00,1.29)	0.11 (0.01,2.07)	0.33 (0.02,7.34)	0.14 (0.00,3.92)	0.07 (0.00,1.38)	0.00 (0.00,0.10)	0.00 (0.00,0.02)	0.02 (0.00,0.79)	0.00 (0.00,0.01)
0.90 (0.04,22.32)	0.00 (0.00,0.16)	0.15 (0.00,5.84)	0.01 (0.00,0.48)	0.00 (0.00,0.24)	0.33 (0.01,8.60)	1.35 (0.06,30.97)	2.72 (0.19,38.11)	GemOxa+Cetuximab	0.55 (0.09,3.42)	0.18 (0.01,3.35)	0.30 (0.02,5.37)	0.91 (0.04,19.07)	0.37 (0.01,10.21)	0.20 (0.01,3.57)	0.01 (0.00,0.26)	0.00 (0.00,0.06)	0.06 (0.00,2.06)	0.00 (0.00,0.03)
1.65 (0.12,22.92)	0.01 (0.00,0.18)	0.27 (0.01,6.52)	0.03 (0.00,0.52)	0.01 (0.00,0.29)	0.60 (0.04,8.93)	2.46 (0.19,31.30)	4.95 (0.74,33.25)	1.82 (0.29,11.35)	GemOxa	0.33 (0.03,3.19)	0.55 (0.06,5.08)	1.65 (0.14,18.87)	0.67 (0.04,10.74)	0.37 (0.04,3.37)	0.02 (0.00,0.26)	0.01 (0.00,0.05)	0.11 (0.01,2.25)	0.00 (0.00,0.02)
4.94 (0.15,158.41)	0.02 (0.00,0.26)	0.82 (0.08,8.30)	0.08 (0.01,0.63)	0.02 (0.00,0.43)	1.81 (0.37,8.96)	7.37 (0.25,221.04)	14.84 (0.77,284.52)	5.46 (0.30,99.80)	3.00 (0.31,28.65)	GemCis+Ramucirumab	1.65 (1.06,2.58)	4.95 (1.63,15.04)	2.01 (0.36,11.34)	1.11 (0.71,1.73)	0.07 (0.02,0.21)	0.02 (0.00,0.41)	0.33 (0.04,2.67)	0.01 (0.00,0.21)
3.00 (0.10,93.95)	0.01 (0.00,0.15)	0.50 (0.05,4.87)	0.05 (0.01,0.37)	0.01 (0.00,0.25)	1.10 (0.23,5.17)	4.47 (0.15,131.03)	9.00 (0.48,168.08)	3.31 (0.19,58.93)	1.82 (0.20,16.78)	0.61 (0.39,0.95)	GemCis+Merestinib	3.00 (1.06,8.49)	1.22 (0.23,6.57)	0.67 (0.54,0.83)	0.04 (0.01,0.12)	0.01 (0.00,0.24)	0.20 (0.03,1.56)	0.01 (0.00,0.12)
1.00 (0.03,35.99)	0.00 (0.00,0.06)	0.17 (0.01,1.99)	0.02 (0.00,0.15)	0.00 (0.00,0.10)	0.37 (0.06,2.30)	1.49 (0.04,50.33)	3.00 (0.14,65.92)	1.10 (0.05,23.17)	0.60 (0.05,6.91)	0.20 (0.07,0.61)	0.33 (0.12,0.94)	GemCis+Durvalumab	0.41 (0.06,2.87)	0.22 (0.08,0.62)	0.01 (0.00,0.06)	0.00 (0.00,0.10)	0.07 (0.01,0.65)	0.00 (0.00,0.05)
2.45 (0.05,112.14)	0.01 (0.00,0.20)	0.41 (0.02,6.82)	0.04 (0.00,0.54)	0.01 (0.00,0.32)	0.90 (0.09,8.68)	3.66 (0.09,157.47)	7.37 (0.26,212.74)	2.71 (0.10,75.06)	1.49 (0.09,23.79)	0.50 (0.09,2.80)	0.82 (0.15,4.40)	2.46 (0.35,17.36)	GemCis+Cediranib	0.55 (0.10,2.91)	0.03 (0.00,0.24)	0.01 (0.00,0.31)	0.17 (0.01,2.30)	0.00 (0.00,0.15)
4.47 (0.14,139.23)	0.01 (0.00,0.23)	0.74 (0.08,7.19)	0.07 (0.01,0.54)	0.02 (0.00,0.38)	1.64 (0.35,7.60)	6.67 (0.23,194.16)	13.43 (0.72,248.79)	4.94 (0.28,87.22)	2.71 (0.30,24.78)	0.90 (0.58,1.42)	1.49 (1.20,1.85)	4.48 (1.62,12.38)	1.82 (0.34,9.67)	GemCis	0.06 (0.02,0.17)	0.02 (0.00,0.36)	0.30 (0.04,2.31)	0.01 (0.00,0.18)
72.95 (2.01,2647.34)	0.24 (0.02,3.01)	12.09 (0.99,147.02)	1.12 (0.13,9.95)	0.32 (0.02,5.07)	26.74 (4.68,152.82)	108.83 (3.20,3702.71)	219.16 (9.90,4853.96)	80.63 (3.81,1706.41)	44.25 (3.84,509.40)	14.77 (4.77,45.70)	24.35 (8.44,70.20)	73.15 (17.12,312.48)	29.74 (4.17,212.21)	16.32 (5.79,46.05)	Gem	0.30 (0.01,7.00)	4.92 (0.50,48.26)	0.15 (0.01,3.51)
244.65 (8.98,6664.04)	0.80 (0.01,45.87)	40.55 (0.95,1721.90)	3.77 (0.10,141.21)	1.08 (0.02,71.41)	89.66 (3.14,2563.92)	364.97 (14.37,9267.57)	734.97 (46.51,11612.93)	270.38 (18.01,4059.50)	148.39 (20.12,1094.31)	49.52 (2.43,1009.45)	81.65 (4.11,1621.93)	245.30 (10.51,5722.68)	99.73 (3.27,3038.64)	54.73 (2.78,1078.93)	3.35 (0.14,78.74)	FUFA	16.49 (0.45,609.21)	0.50 (0.19,1.30)
14.84 (0.27,806.92)	0.05 (0.00,1.47)	2.46 (0.12,51.97)	0.23 (0.01,4.14)	0.07 (0.00,2.35)	5.44 (0.42,69.61)	22.14 (0.43,1136.10)	44.58 (1.27,1565.59)	16.40 (0.49,553.67)	9.00 (0.45,181.95)	3.00 (0.37,24.14)	4.95 (0.64,38.34)	14.88 (1.53,144.72)	6.05 (0.44,84.11)	3.32 (0.43,25.41)	0.20 (0.02,2.00)	0.06 (0.00,2.24)	FOLFIRINOX	0.03 (0.00,1.12)
492.65 (17.95,13522.75)	1.62 (0.03,92.95)	81.65 (1.91,3490.87)	7.60 (0.20,286.34)	2.18 (0.03,144.68)	180.55 (6.27,5202.06)	734.95 (28.72,18809.00)	1480.00 (92.81,23600.70)	544.46 (35.93,8251.45)	298.81 (40.01,2231.70)	99.73 (4.85,2049.86)	164.43 (8.21,3293.84)	493.96 (21.00,11616.69)	200.83 (6.54,6164.38)	110.22 (5.54,2191.16)	6.75 (0.29,159.84)	2.01 (0.77,5.29)	33.20 (0.89,1235.40)	BSC

GemCis: gemcitabine plus cisplatin; GemOxa: gemcitabine plus oxaliplatin; GemS1: gemcitabine plus S-1; S1Cis: S1 plus cisplatin; XELOX: capecitabine plus oxaliplatin; BSC: best supportive care; FUFA: fluorouracil+folinic; FOLFIRINOX: oxaliplatin plus irinotecan plus infusional fluorouracil.

**Table 5:** Surface under the cumulative ranking curve values for progression-free survival.

Treatment	SUCRA
GemOxa+Erlotinib	91.2
GemCis+Durvalumab	82.7
GemOxa+Panitumumab	81.2
GemOxa+Cetuximab	79
XELOX	76
GemOxa	69.5
GemCis+Cediranib	66
GemCis+Merestinib	64.2
GemS1	63.7
GemCis	51.9
S1Cis	50.5
GemCis+Ramucirumab	49
FOLFIRINOX	37.1
S1	22.5
Gem	21.6
FUFA	13.9
Gem+Vandetanib	13.3
Vandetanib	10.5
BSC	6.2

GemCis: gemcitabine plus cisplatin; GemOxa: gemcitabine plus oxaliplatin; GemS1: gemcitabine plus S-1; S1Cis: S1 plus cisplatin; XELOX: capecitabine plus oxaliplatin; BSC: best supportive care; FUFA: fluorouracil+folinic; FOLFIRINOX: oxaliplatin plus irinotecan plus infusional fluorouracil.

## Data Availability

The original contributions presented in the study are included in the article; further inquiries can be directed to the corresponding author.
